This article has been retracted.

# Decreased Polymorphonuclear Myeloid-Derived Suppressor Cells and ROS Production Correlated Closely with Bronchopulmonary Dysplasia in Preterm Infants

**DOI:** 10.1155/2022/9010354

**Published:** 2022-09-20

**Authors:** Wangkai Liu, Sitao Li, Yushan Li, Wei Shen, Haitian Chen, Xiaoyu Li, Linnuan Cai, Fan Wu, Yumei Liu, Qiong Meng, Xiaoyun Jiang

**Affiliations:** ^1^Department of Pediatrics, The First Affiliated Hospital, Sun Yat-sen University, Guangzhou, China; ^2^Department of Pediatrics, The Sixth Affiliated Hospital, Sun Yat-sen University, Guangzhou, China; ^3^Department of Pediatrics, Southern Medical University, Guangzhou, Guangdong, China; ^4^Department of Obstetrics, The First Affiliated Hospital, Sun Yat-sen University, Guangzhou, China; ^5^Department of Pediatrics, Third Affiliated Hospital, Guangzhou Medical University, Guangzhou, China; ^6^Department of Neonatology, Guangdong Provincial People's Hospital, Guangdong Academy of Medical Sciences, Guangzhou, China; ^7^Department of Pediatrics, Guangdong Second Provincial General Hospital, Guangzhou, China

## Abstract

**Background:**

Bronchopulmonary dysplasia (BPD) is one of the most serious complications in premature infants. Myeloid-derived suppressor cells (MDSCs) have been indicated to promote immune tolerance and induce anti-inflammatory responses during the neonatal stage. However, the role of MDSCs in BPD has not been completely expounded.

**Methods:**

130 cases of newborns were collected from six tertiary hospitals in Guangzhou from August 2019 to June 2022. They were divided into BPD group, non-BPD preterm infants group, and term infants group according to gestational age and presence of BPD. The peripheral blood was collected and used to analyze the proportion, phenotypic, and function of MDSCs at 3 to 7 days and 8 to 14 days after birth, respectively.

**Results:**

We indicated that the number of both MDSCs in premature infants is reduced, and the number of polymorphonuclear myeloid-derived suppressor cells (PMN-MDSCs) in peripheral blood of BPD infants was significantly lower than that of non-BPD infants under 34 weeks of gestational age (*P* < 0.05). Furthermore, PMN-MDSCs from peripheral blood of patients presented inhibitory effect on proliferation of CD4^+^T and CD8^+^T cells in each group. However, PMN-MDSCs from BPD group had obviously weaker inhibitory effect on proliferation of CD4^+^T and CD8^+^T cells than that from non-BPD preterm infants group. In addition, we demonstrated that the expression of NADPH oxidase (Nox2) and reactive oxygen species (ROS) in PMN-MDSCs of BPD children was significantly lower than that in non-BPD preterm infants, suggesting that ROS pathway was affected in BPD in premature infants.

**Conclusion:**

This study preliminarily revealed the role of PMN-MDSCs in the pathogenesis of BPD in premature infants. The specific immune regulation mechanism of PMN-MDSCs in BPD will provide new ideas and strategies for clinical prevention and treatment of BPD in premature infants.

## 1. Introduction

Preterm birth is not only a common but also a serious disease of newborns with a second-highest mortality rate among children under five [1]. Studies have shown that BPD is the most prevalent short-term complication of preterm infants [2]. In a study for newborns with a gestational age of 24 to 31 weeks and a birth weight of less than 1500 g in 11 high-income countries indicated that although mortality in early preterm infants decreased in most countries, the incidence of BPD increased [3]. An analysis of the short-term outcomes of very preterm infants after the discharge from Guangdong Province, China, showed that the neonatal survival rate increased from 36.2% in 2008 to 59.3% in 2017, and the incidence of BPD also significantly increased by more than 50% [4].

MDSCs are a heterogeneous group of cells which have a strong immune inhibitory function [5]. MDSCs are divided into two types according to the expression of surface antigens, including PMN-MDSCs and monocytic MDSCs (M-MDSCs) [6]. M-MDSCs mainly inhibit the function of T cells in an antigen-nonspecific manner by increasing the activity of arginase, while PMN-MDSCs inhibit T cell responses in an antigen-specific manner typically using ROS as immune mediators [7].

Immunosuppression is a major feature of MDSCs, and T cells are their primary targets. Previous studies have shown that MDSCs exert their immunosuppressive effects by regulating multiple pathways, such as regulatory T cell (Treg), iNOS and ARG1, ROS, and peroxynitrite (ONOO^−^) pathways [8]. In our previous research, we found that the oxygen stress pathway related genes were significantly up-regulated in lung tissue, and the transcription of glutathione S-transferase alpha 2 (Gsta2) was also significantly increased in a lung transcriptomic data with an early in the disease course of mouse BPD model. The results suggested that oxygen damage might be one of the important factors that cause early lung inflammation. More importantly, we observed that the MDSCs marker genes S100A8 and S100A9 were significantly down-regulated (unpublished data). We also revealed that MDSCs were significantly deficient in quantity, function, and antibacterial activity in preterm mice, compared with the term mice, suggesting that MDSCs had a protective effect on the development of inflammation in neonatal mice [9].

Taken together, these findings proved that BPD posed a great threat to the quality of life of premature infants. However, its pathogenesis is not fully elucidated. In addition, inflammatory response is an important factor in the development of BPD. It is necessary to find new immune regulation mechanisms related to inflammation to prevent and treat BPD. MDSCs were proved to play an important immunosuppressive role in the early neonatal period and protect the body from anti-inflammatory and anti-infective effects. Thus, this study aims to explore the function of MDSCs in the development of BPD.

## 2. Materials and Methods

### 2.1. Human Subjects

Neonatal cases born in the neonatology department of 6 tertiary hospitals (The First Affiliated Hospital of Sun Yat-sen University, Nanfang Hospital, Guangdong Provincial People's Hospital, Guangdong Second Provincial General Hospital, the Third Affiliated Hospital of Guangzhou Medical University, the Sixth Affiliated Hospital of Sun Yat-sen University) in Guangzhou were collected from August 2019 to June 2022. The inclusion criteria include preterm infants and term infants not included in the exclusion criteria. They were divided into BPD group, non-BPD premature infants group, and non-BPD term infants group based on their gestational age and presence of BPD. The peripheral blood from all cases was collected at 3-7 days and 8-14 days after birth. 30 premature infants with BPD were collected. In order to analyze the relationship between the occurrence of BPD and the existence of MDSCs, preterm infants and term infants with the same gestational age and sampling age without BPD were collected in a ratio of 1 : 1 : 1 as the control group. Exclusion criteria include congenital heart disease (atrial septal defect, ASD; ventricular septal defect, VSD; and patent ductus arteriosus, PDA), persistent pulmonary hypertension in the neonate (PPHN), severe congenital malformations, chromosomal abnormalities, genetic metabolic diseases, anemia, and cases with incomplete data. This project had obtained the ethical exemption of Clinical Research and Animal Trials of the First Affiliated Hospital of Sun Yat-sen University ethics committee (No. [2020]521).

#### 2.1.1. Collected Data

According to the 2001 NICHD diagnostic criteria, 30 premature infants with BPD were collected, and the preterm infants and term infants without BPD with the same gestational age were collected as the control group at a ratio of 1 : 1 : 1, with total of 90 cases.

#### 2.1.2. Analyzing the Proportions and Phenotypes of MDSCs by Flow Cytometry

In order to clarify whether MDSCs can be used as an important predictor of BPD, the correlation analysis was carried out between the levels of MDSCs subtypes and the main indicators related to BPD disease.

#### 2.1.3. Analyzing the Function of MDSCs in BPD

The PMN-MDSCs of 5 BPD patients and 5 non-BPD patients were sorted by flow cytometry. Their PMN-MDSCs were co-cultured with CD4^+^/CD8^+^ T cells to detect the effect of PMN-MDSCs on the T cell proliferation; In order to figure out whether the PMN-MDSCs of BPD children had immunosuppressive function defects, RT-qPCR was used to detect PMN-MDSCs function-related genes (Arg1, Nos2, and Nox2) and anti-inflammatory factors (IL-10, TGF-*β*, and IFN-*γ*) in 10 BPD children and 10 non-BPD children.

### 2.2. In Vitro Culture of Peripheral Blood MDSCs

0.5 ml peripheral blood from patients was collected and the erythrocytes were lysed. Then, it was washed with pre-cooled RPMI medium and resuspended for counting. The cell suspension was laid on 48-well plates at a density of 1 × 10^6^ per well or 2-2.5 × 10^6^ in 24-well plates. 20 ng/mL human GM-CSF and 20 ng/mL IL-6 were added in the plates to induce the differentiation of cells into human MDSCs. After 3 days of culture, 80% fluid was changed, and phenotypic analysis or functional test was performed until 6 days of culture.

### 2.3. Flow Cytometry and Sorting

Cells (1 × 10^6^ cells) were resuspended in 4 ml 1 × phosphate buffer saline (PBS) in a 5 ml centrifuge tube then centrifuged at 4, 300 rmp/min for 5 min. The supernatant was discarded and then the cells were stained with 100 *μ*L antibody (1 : 400 dilution) at 4°C for 30 min in dark. Then, cells were diluted in PBS to a total volume of 4 ml and centrifuged at 4,300 rmp/min for 5 min. The cells were resuspended with 500 *μ*L 1 × PBS and were analyzed by flow cytometry. Briefly, cells were stained with surface markers HLA-DR, CD1b, CD14, CD15, and LOX-1. The gating strategy for PMN-MDSCs was CD11b^+^HLA-DR^−^CD15^+^CD14^−^ or CD15^+^LOX-1^+^. The proportion of PMN-MDSC cells was detected and sorted by flow cytometry.

### 2.4. Co-Culture of MDSC and T Cells

Labeled CD3^+^ T cells were labeled with carboxyfluorescein succinimidyl amino ester (CFSE, 1*μ*M) and were co-cultured at different ratios (8 : 1, 4 : 1, and 2 : 1) with PMN-MDSCs from all the groups in U-bottomed 96-well plate and stimulated with anti-CD3 and anti-CD28 for 3 days. Then, the CD4^+^ and CD8^+^ T cells were stained and detected CFSE with FITC panel [10].

### 2.5. Peripheral Blood Mononuclear Cell (PBMC) Isolation and ROS Analysis

PBMCs were isolated from whole blood by Ficoll centrifugation and analyzed immediately according to the previous report [11]. Then, cells were incubated with anti-human fluorescence-conjugated antibodies (CD11b-BUV396, HLA-DR-APC-cy7, CD14-APC, and CD15-BV605). And then intracellular ROS levels were determined using dichlorodihydrofluorescein diacetate (DCFH-DA) (Invitrogen). Briefly, cells that were pre-treated with different reagents were incubated with 20 *μ*M DCFH-DA in Hanks' balanced salt buffer for 30 min at 37°C. The ROS level was quantified using a FACS flow cytometer ((BD LSR fortessa, BD Biosciences, San Jose, CA, USA).

### 2.6. Statistical Analysis

Statistical analysis was performed with GraphPad Prism version 5.0a and SPSS 22.0. The statistical data are presented as means ±standard deviation (SD). Differences between two groups were evaluated by Student's *t*-test. *P* values < 0.05 were considered significant.

## 3. Results

A total of 130 infants were enrolled actually. We collected only 23 patients with BPD, and 107 patients (75 preterm infants and 32 term infants) without BPD. There was no gender difference.

### 3.1. Correlation between MDSCs and BPD

#### 3.1.1. Distribution of MDSCs by Gestational Age

As shown in Figure 1(a), in the absence of infection, BPD premature infants with gestational ages (GA) <28 weeks had lower M-MDSCs (CD11b^+^HLA^−^DR^−^CD14^+^CD15^−^) and PMN-MDSCs (CD11b^+^HLA^−^DR^−^CD14^−^CD15^+^) levels than that in premature infants with GA >28 weeks. Furthermore, the proportion of CD15^+^LOX-1^+^ in peripheral blood of late preterm infants with 34-37 weeks GA was significantly higher than that of preterm infants born at 28-32 weeks of GA (*P* =0.0026). However, compared with preterm infants with 32-34 weeks GA, the proportion of CD15^+^LOX-1^+^ in peripheral blood of late preterm infants with 34-37 weeks GA was significantly increased (*P* =0.008). These results suggested that the smaller gestational age might contribute to the smaller number of MDSCs, with predominant decrease in PMN-MDSCs.

#### 3.1.2. Comparative Analysis of MDSCs with Different Phenotypes in Preterm Infants Less Than 34 Weeks Gestational Age

Since almost all BPD infants in this study had a gestational age <34 weeks, there would be a greater bias if compared with term infants or preterm infants > 34 weeks GA. Thus, statistical analysis was carried out for the control group with GA <34 weeks between the infants with or without infection at different blood sampling time points, etc.

The results showed that there was no difference in the proportion of M-MDSCs (CD11b^+^HLA^−^DR^−^CD14^+^CD15^−^), CD15^+^LOX1^+^, and PMN-MDSCs (CD11b^+^HLA^−^DR^−^CD14^−^CD15^+^) between premature infants with infection (3-7d after birth, GA <34w) and preterm infants with BPD (3-7d after birth, GA <34w) at the same period (*P* > 0.05) (Figure 1(b)). However, the proportion of PMN-MDSCs (CD11b^+^HLA^−^DR^−^CD14^−^CD15^+^) in peripheral blood of children with BPD was significantly lower than that in premature infants without BPD and infection (3-7d after birth, GA <34w) (*P* < 0.05). The proportion of CD15^+^LOX-1^+^ and M-MDSCs (CD11b^+^HLA^−^DR^−^CD14^+^CD15^−^) in BPD children also had a downward trend without statistical significance (Figure 1(c)).

The proportion of PMN-MDSCs (CD11b^+^HLA^−^DR^−^CD14^−^CD15^+^), CD15^+^LOX-1^+^, and M-MDSCs (CD11b^+^HLA^−^DR^−^CD14^+^CD15^−^) in peripheral blood of premature was not significantly different between infants without BPD and infection (8-14d after birth, GA <34w) and premature infants with BPD (*P* > 0.05) (Figure 1(d)). Compared with non-BPD preterm infants with infection, both the proportion of M-MDSCs and CD15^+^LOX-1^+^ cells of BPD infants with infection (8-14d after birth, GA <34w) increased (Figure 1(e)), and the proportion of PMN-MDSCs decreased without statistical significance (*P* > 0.05).

These data suggested that the decrease of PMN-MDSCs may lead to the suppression of their immune function which will affect BPD development.

### 3.2. Analysis of PMN-MDSCs Function in Infants with BPD

#### 3.2.1. Functional Analysis of PMN-MDSCs Inhibiting the Proliferation of CD4^+^/CD8^+^ T Cells

To determine whether MDSCs in preterm infants have an immunosuppressive function and whether there is a defect in the immunosuppressive function of MDSCs in BPD patients, the function of MDSCs was detected. Peripheral blood PMN-MDSCs of BPD infants were sorted and co-cultured with T cells at 2 : 1, 4 : 1, and 8 : 1, while PMN-MDSCs of non-BPD term infants group and non-BPD preterm infants group were co-cultured with T cells as a control group.

Flow cytometry was used to detect the effect of PMN-MDSCs on CD4^+^ T cell proliferation. The results in Figure 2(a) showed that, regardless of the ratio,, CD4^+^ T cells proliferation in BPD group was remarkably higher than that in non-BPD term infants group (*P* < 0.01) when CD4^+^ T cells and PMN-MDSCs were co-cultured. Similarly, when CD4^+^ T cells and PMN-MDSCs were co-cultured in the ratio of 2 : 1, 4 : 1, and 8 : 1, the CD4^+^ T cells proliferation in BPD group was significantly higher than that in non-BPD preterm infants group (*P* < 0.05, *P* < 0.01). The peripheral blood PMN-MDSCs of all the children in each group had an inhibitory effect on the CD4^+^ T cells proliferation. However, the inhibition was apparently weaker in the BPD premature infants group than that in the non-BPD preterm infants group, consistent with the reduced proportion of its flow phenotype.

For CD8+ T cells, the results in Figure 2(b) showed that the CD8^+^ T cells multiplication of BPD preterm infant group was markedly higher than that of non-BPD term infants group (*P* < 0.05) when CD8^+^ T cells were co-cultured with PMN-MDSCs at 8 : 1. The propagation of CD8^+^ T cells showed the similar result when co-cultured at 4 : 1 (*P* < 0.01) and 2 : 1 (*P* < 0.01). The proliferation of CD8^+^ T cells in the BPD preterm infants group was significantly higher than that in the non-BPD preterm infant group (*P* < 0.05) when CD8^+^ T cells and PMN-MDSCs were co-cultured at 2 : 1. However, there was no statistical significance when CD8^+^ T cells were co-cultured with PMN-MDSCs at a ratio of 8 : 1 and 4 : 1 (*P* > 0.05). The PMN-MDSCs of all groups suppressed the proliferation of CD8^+^ T cells. Compared with the two other groups, the inhibitory effect was significantly weaker in BPD group, consistent with the reduced proportion of its flow phenotype. These results suggested that although the number of PMN-MDSCs from children with BPD did not decrease, the ability of CD4^+^/CD8^+^ T cells proliferation suppression was attenuated.

### 3.3. Screening and Validation of Molecules Related to MDSCs Immunosuppressive Function

#### 3.3.1. Expression of Arg1, Nos2, and Nox2 in PMN-MDSCs

The expressions of three classical molecules related to the immunosuppressive function of MDSCs were detected by qRT-PCR, including arginase 1 (Arg1), inducible nitric oxide synthesis (Nos2 or iNos), and Nox2. The results showed that the expression of Arg1 and Nos2 in PMN-MDSCs of BPD infants was not significantly different from that of non-BPD cases. However, the expression of Nox2 in PMN-MDSCs of BPD cases was obviously lower than non-BPD cases (*P* < 0.05) (Figure 3(a)), indicating that PMN-MDSCs have a certain immunosuppressive function in BPD children and the defect was manifested in the low expression of Nox2.

#### 3.3.2. Expression of IL-10, TGF-*β*, and IFN-*γ* in PMN-MDSCs

The expression of PMN-MDSCs immunosuppressive function-related cytokines IL-10, TGF-*β*, and IFN-*γ* in BPD and non-BPD premature infants was also detected by RT-qPCR. Compared with non-BPD premature infants, the expressions of IL-10 and TGF-*β* were significantly lower in PMN-MDSCs of BPD children (*P* < 0.05). In contrast, the expression of IFN-*γ* in PMN-MDSCs of BPD children also showed a downward trend, but did not meet statistical significance (*P* > 0.05) (Figure 3(b)).

### 3.4. Comparative Analysis of ROS Levels of BPD and Non-BPD Preterm Infants

ROS levels were measured in the peripheral blood of 14 preterm infants aged 2 to 7 days. They were then grouped according to whether they were diagnosed with BPD at 28 days old. The result showed that ROS level in the peripheral blood from non-BPD preterm infants was significantly higher than that in the BPD infants (*P* < 0.05) (Figure 4).

## 4. Discussion

MDSCs are a class of pathologically activated immature myeloid cells with potent immunosuppressive functions [11, 12]. Recent studies have shown that MDSCs are important to the induction of physiological immune tolerance which could induce individual airway tolerance and prevent asthma attacks [13, 14]. MDSCs have also been found to promote maternal-fetal tolerance and ensure the normal progression of pregnancy [15, 16]. Besides, MDSCs level at birth can predict necrotizing enterocolitis in premature infants [9]. However, whether PMN-MDSC levels are different in peripheral blood of BPD and non-BPD children and whether it can be used as a diagnostic marker of BPD remains unclear. In the present study, we demonstrated that the number of MDSCs reduced in preterm infants, and on the premise of zero infections in preterm infants with GA <34w, the number of PMN-MDSCs from BPD children at 3-7 days after birth was obviously lower than that from non-BPD group. However, there was no statistical difference in the number of PMN-MDSCs, M-MDSCs, and LOX-1 between BPD group and non-BPD group in other groups, especially for sampling time point at 8-14d after birth. These results indicated that BPD might be mainly related to the rapid decline of MDSCs about 10 days after birth.

Co-cultured CD4+ T cells and CD8+ T cells with PMN-MDSCs assay is a classic experiment to judge whether the function of MDSCs is defective. Therefore, we speculated that if PMD-MDSCs from the peripheral blood of BPD group have functional defects, the proliferation of CD4+T and CD8+T cells may also be affected indirectly. In this study, we demonstrated that PMN-MDSCs derived from BPD infants had significantly weaker inhibitory effects on the proliferation of both CD4+ T and CD8+T cells than that derived from the non-BPD premature infants. This finding indicated that there was a certain defect in the immune function of PMN-MDSCs in children with BPD. To be specific, PMN-MDSCs were incapable of taking anti-inflammatory and protective effects and further resulted in the persistence of inflammation, which in turn led to the occurrence and development of BPD.

MDSCs exert immunosuppressive function via regulating multiple pathways. To further verify the specific pathway MDSCs involved in, the expression of three classical molecules related to the immunosuppressive function of MDSCs was detected, including Arg1, Nos2, and Nox2. The results showed that the expressions of Nox2 in PMN-MDSCs from BPD group were significantly lower than that of non-BPD preterm infants group. In contrast, there was no significant difference between BPD group and non-BPD preterm infants group for the expressions of Arg1 and Nos2 in PMN-MDSCs. This result indicated that ROS pathway, as an important pathway for MDSCs to exert immunosuppressive functions, was affected. In addition, we found that ROS level of BPD infants was significantly lower than that of non-BPD preterm infants group, which prompted that low ROS level in first 7 days of life may predict the development of BPD. These results were consistent with the findings reported by Corzo et al. [17] that MDSCs can promote the expression of NOX2 to generate a large amount of ROS, which is considered to be an inhibitor of tumor antigen-specific T cells [17] . In addition, we speculated that low ROS level might be a signal to implement clinical intervention to prevent BPD.

Inflammation is an important factor in the pathogenesis of BPD. MDSCs could affect the function of other immune cells to exert its immunosuppressive and anti-inflammatory effects through secreting anti-inflammatory factors like IL-10 and TGF-*β* [18]. Our results showed that the expressions of IL-10 and TGF-*β* in PMN-MDSCs derived from BPD group were significantly lower than non-BPD preterm infants group, suggesting that the ability to secrete anti-inflammatory cytokines is also decline in peripheral blood PMN-MDSCs of BPD infants with a certain functional defect. These results indicated that the anti-inflammatory effects of PMN-MDSCs were suppressed in premature infants. In addition, our previous study found that lung oxygen damage occurs in the early stage of BPD, and the oxygen stress protein arachidonic acid 15 lipoxygenase (ALOX15) is significantly up-regulated in the early stage of BPD, which catalyzes the production of oxidized low-density lipoprotein (oxLDL) (unpublished data). oxLDL can mediate apoptosis through its receptor LOX-1 which is a signature protein of MDSCs, suggesting that ALOX15 may act on the occurrence of BPD by regulating MDSCs. Based on these findings, we will further validate the scientific hypothesis through in vitro and in vivo experiments which will hopefully reveal new immune mechanisms in the pathogenesis of BPD and provide new strategies for the clinical treatment of BPD.

In addition, there remain several limitations for the current study. First, although several accurate trends are proven, some statistically significant difference was not observed due to a relative low sample size. Second, some potential influencing factors like birth weight and prophylactic antibiotic use should be included. Third, the specific immunosuppressive function and mechanism of MDSCs in BPD should be verified by establishing BPD animal model for allogeneic intervention.

In conclusion, we revealed that the number of PMN-MDSCs and the levels of anti-inflammatory factors in peripheral blood of BPD premature infants early after birth were significantly lower than those of non-BPD infants, with a defective immunosuppressive function. Besides, we indicated that low ROS level in early postnatal days may be a potential predictor of BPD. These findings suggested that PMN-MDSCs participated in the pathogenesis of BPD in premature infants via regulating the ROS pathway. Our study preliminarily revealed the role of PMN-MDSCs in the pathogenesis of BPD. However, the specific mechanism still needs to be further studied and validated.

## Figures and Tables

**Figure 1:** Quantification of M-MDSCs, PMN-MDSCs, and LOX-1 in peripheral blood. (a) Quantification of M-MDSCs, PMN-MDSCs, and LOX-1 in peripheral blood of infants (3-7d after birth, without infection) at GA<28 W (*n* =3), GA 28~32 W (*n* =16), GA 32~34w (*n* =14), GA 34~37w (*n* =6), and GA >37w (*n* =21) (^∗∗^, *P* < 0.01) (^∗∗∗^, *P* < 0.001). (b) The proportion of M-MDSCs, PMN-MDSCs, and LOX-1 in peripheral blood of children with BPD (*n* =17) and without BPD (3-7d after birth, gestational age <34w, with infection) (*n* =36). (c) Quantification of M-MDSCs, PMN-MDSCs, and LOX-1 in peripheral blood of children with BPD (*n* =7) and without BPD (3-7d after birth, gestational age <34w, without infection) (*n* =49) (^∗^, *P* < 0.05). (d) The proportion of M-MDSCs, PMN-MDSCs, and LOX-1 in peripheral blood of children with BPD (*n* = 4) and without BPD (8-14d after birth, gestational age <34w, without infection) (*n* = 11). (e) The proportion of M-MDSCs, PMN-MDSCs, and LOX-1 in peripheral blood of children with BPD (*n* = 1) and without BPD (8-14d, after birth gestational age <34w, with infection) (*n* =14) (^∗^, *P* < 0.05).

**Figure 2:** PMN-MDSCs inhibited the proliferation of CD4^+^/CD8+ T cells. (a) The proliferation rate of CD4^+^ cells was detected by flow cytometry after 3 days. CD4^+^ cells and PMN-MDSCs were co-cultured in different proportions. The figure above is typical flow chart and the figure below is statistical chart. PMN-MDSCs inhibited the proliferation of CD8^+^ T cells (*n* = 11) (^∗^*P* < 0.05, ^∗∗^*P* < 0.01). (b) Flow cytometry was used to detect the proliferation rate of CD8^+^ cells after 3 days. CD8^+^ T cells and PMN-MDSCs were co-cultured in different proportions. The figure above is typical flow chart and the figure below is statistical chart (*n* = 11) (^∗^*P* < 0.05, ^∗∗^*P* < 0.01).

**Figure 3:** Expression of PMN-MDSCs immunosuppressive function-related three classical molecules and cytokines. (a) Expression of Arg1, Nos2, and Nox2 in PMN-MDSCs was detected by RT-qPCR (*n* =3 per group) (^∗^*P* < 0.05). (b) Expression of IL-10, TGF-*β*, and IFN-*γ* in PMN-MDSCs was detected by RT-qPCR (*n* =3 per group) (^∗^*P* < 0.05).

**Figure 4:** ROS levels in BPD infants and non-BPD preterm infants (control, *n* = 9; BPD, *n* = 5) (^∗^, *P* < 0.05).

## Data Availability

The data used to support the findings of this study are included within the article and figure files.
